# Effects of Serum LDL-C, CysC, and D-D in Patients with Coronary Atherosclerotic Heart Disease

**DOI:** 10.1155/2022/5771960

**Published:** 2022-06-28

**Authors:** Chaofeng Shen, Jing Wang, Sijia Tu

**Affiliations:** ^1^Department of Cardiovascular Medicine, First People's Hospital of Linping District, Hangzhou 311100, Zhejiang, China; ^2^Department of Ultrasound, Fifth People's Hospital of Linping District, Hangzhou 311100, Zhejiang, China

## Abstract

**Objective:**

To investigate the effects of low-density lipoprotein cholesterol (LDL-C) and serum cystatin C (CysC) combined with D-dimer (D-D) on patients with coronary atherosclerotic heart disease (CHD).

**Methods:**

90 patients with CHD who were admitted to our hospital and diagnosed by coronary angiography (CAG) from February 2020 to June 2021 were selected as the study subjects. 90 patients were grouped according to different types and branches of coronary lesions, and 30 patients with outpatient health check-ups at the same period were selected as the control group, and the differences in serum LDL-C, CysC, and D-D levels between the groups were compared. The logistic regression model was built to explore risk factors affecting the occurrence of CHD. Also, receiver operating characteristic (ROC) curves were drawn to analyze the diagnostic value of LDL-C, CysC, and D-D in CHD.

**Results:**

In the comparison of LDL-C, CysC, and D-D levels, CHD group > control group (*P* < 0.05); stable angina (SAP) group > unstable angina (UAP) group > acute myocardial infarction (AMI) group (*P* < 0.05); three-branch group > two-branch group > single-branch group (*P* < 0.05). The logistic regression model showed that high expression levels of LDL-C, CysC, and D-D, male gender, and combined hypertension were risk factors for CHD. The area under the curve (AUC) of the combination of LDL-C, CysC, and D-D was 0.868, and the sensitivity and specificity were 88.89% and 73.33%, respectively, which are higher than those in single diagnosis (*P* < 0.05).

**Conclusions:**

LDL-C, CysC, and D-D are highly expressed in CHD samples, and the combination of the three is beneficial to enhance the diagnostic accuracy of clinical CHD.

## 1. Introduction

Coronary atherosclerotic heart disease (CHD) has no obvious symptoms in the early stage, and the onset is more acute. Most patients are admitted to hospital due to acute myocardial infarction or sudden cardiac death, which is life-threatening [1, 2]. Therefore, it is of great significance to accurately diagnose and evaluate the degree of coronary artery disease in cases with CHD. Although coronary angiography is the gold standard for evaluating the severity of CHD, it has inevitable limitations as a high-cost, invasive procedure [3]. Studies have found that dyslipidemia is closely connected with CHD, and low-density lipoprotein cholesterol (LDL-C) is a crucial hazardous factor for CHD [4]. Meanwhile, serum cystatin C (CysC) can better predict the danger of cardiovascular events in high-risk patients than creatinine or glomerular filtration rate [5]. D-Dimer (D-D) is a unique product of secondary fibrin hyperdegradation. An abnormal increase in the level of D-D in humans indicates that the body is in a hypercoagulable state and a secondary hyperfibrinolysis state. Its serum content is important in the diagnosis of thrombotic diseases. It is of great significance in terms of prognosis and judgment [6]. At present, there are few reports on the relationship between CHD and LDL-C, CysC, and D-D. In this study, the levels of LDL-C, CysC, and D-D were measured in patients with CHD, with the aim of investigating the effects of these indicators on CHD patients and providing new serum biomarkers for the diagnosis of CHD.

## 2. Subjects and Methods

### 2.1. Clinical Information

Research objects: 120 patients hospitalized in our hospital from February 2020 to June 2021 were collected. Another 30 cases with outpatient health check-ups during the same period were selected as the control group. The study was approved by the Hospital Ethics Committee. A flowchart of patient selection and classification is shown in Figure 1.

Inclusion criteria were as follows:

1. To be diagnosed with CHD.
2. At least one artery (left main stem, left anterior descending branch, gyral branch, and coronary artery) and/or ≥50% reduction in the internal diameter of any 1 of the small branches of the vessel as confirmed by coronary angiography (CAG).
3. To be cognitively and mentally normal.
4. Know and agree to this study.

Exclusion criteria were as follows:

1. With malignant tumor.
2. With valvular heart disease or cardiomyopathy.
3. Active rheumatic disease.
4. Severe thyroid disease.
5. Recent history of taking glucocorticoids.

### 2.2. CAG Examination

All CAG examinations are carried out by doctors with ≥5 years of experience in cardiovascular intervention. Based on CAG findings, there were 34 single-branch lesions, 30 double-branch lesions, and 26 triple-branch lesions in this study. According to clinical symptoms, electrocardiogram, and serum enzymatic changes, they were divided into 25 cases of stable angina pectoris (SAP), 30 cases of unstable angina pectoris (UAP), and 35 cases of malformed myocardial infarction (AMI).

### 2.3. Data Collection

Gender, age, smoking, and disease history of each enrolled patient were routinely recorded. Under the normal diet of the patient, they were required to fast for 10 hours overnight, and then fasting peripheral venous blood was collected the next morning to measure fasting blood glucose (FBG), blood urea nitrogen (BUN), creatinine (Cr), total cholesterol (TC), triglyceride (TG), LDL-C, CysC, and D-D.

### 2.4. Statistical Methods

SPSS20.0 software was used to analyze the data. Enumeration data were conducted with Pearson's *χ*^2^ test, and the *T*-test was used for measurement data. Logistic regression models were established to explore the risk factors affecting the occurrence of CHD, and the receiver operating characteristic (ROC) curve was drawn to analyze the diagnosis value of LDL-C, CysC, and D-D in CHD. The inspection level is *α* = 0.05.

## 3. Results

### 3.1. Comparison of General Clinical Data of Patients with Various Clinical Kinds of CHD

As shown in Table 1, both gender and hypertension had significant differences in two groups with different clinical types (*P* < 0.05).

### 3.2. Relationship between the Number of Different Lesions in Patients with CHD and General Clinical Data

In Table 2, our research showed that gender and hypertension showed significant differences between the controls and cases with different lesion counts (*P* < 0.05).

### 3.3. Comparison of LDL-C, CysC, and D-D Levels between Cases and Controls

The contents of LDL-C, CysC, and D-D in cases were higher than those in controls (*P* < 0.05) (Table 3).

### 3.4. Comparison of LDL-C, CysC, and D-D Levels in Patients with Various Clinical Types of CHD

The levels of LDL-C, CysC, and D-D (Table 4 and Figures 2–4) in the SAP group, UA group, and AMI group were increased in turn (*P* < 0.05).

### 3.5. Comparison of LDL-C, CysC, and D-D Levels in CHD Patients with Different Lesion Counts

The levels of LDL-C, CysC, and and D-D were the highest in the three-vessel group and the lowest in the single-vessel group (*P* < 0.05) (see Table 5 and Figures 5–7).

### 3.6. Analysis of Risk Factors Affecting the Occurrence of CHD

In Table 6, a logistic regression model was established with the occurrence of CHD as the dependent variable and serum LDL-C, CysC, and D-D expression levels, male gender, and combined hypertension as independent variables. High expression levels of LDL-C, CysC, and D-D, male gender, and combined hypertension were risk factors for CHD (*P* < 0.05).

### 3.7. Analysis of the Diagnostic Efficacy of LDL-C, CysC, and D-D in CHD

As shown in Table 7 and Figure 8, the AUC of LDL-C, CysC, and D-D combined diagnosis of CHD was 0.868, and the sensitivity and specificity were 88.89% and 73.33%, respectively, which were higher than those in single diagnosis (*P* < 0.05).

## 4. Discussion

CHD presents a younger onset trend due to the influence of improper diet, excessive smoking and drinking, lack of exercise, and other factors [7]. Percutaneous coronary intervention (PCI) is a common and important method for CHD treatment, which can visually display the degree of coronary stenosis during the operation. However, not all CHD patients accept PCI due to objective factors such as economic burden and medical configuration. Therefore, many scholars have been looking for reliable serological indicators that can reflect coronary conditions for clinical diagnosis, so as to provide better management and prevention of CHD patients [8].

Most of the cholesterol in the human body exists and is transported in the form of binding to lipoproteins and then transported to various parts of the body to play corresponding roles [3]. Studies have shown that the elevated contents of total cholesterol and LDL-C in the blood circulation are related to coronary atherosclerosis [9]. Monitoring LDL-C level is the core strategy of the guidelines for the treatment of dyslipidemia at home and abroad [10]. Dyslipidemia accelerates the process of atherosclerosis, and LDL-C is the main factor causing damage to vascular endothelial cells and vascular smooth muscle cells. Serum CysC is not disturbed by gender, diet, and muscle mass and is a sensitive indicator of renal function [11]. At the same time, CysC may be involved in atherosclerotic vascular disease by affecting extracellular matrix degradation, vascular wall remodeling, inflammatory response, and other processes [12]. Various coagulation factors and platelets have always been involved in the occurrence of CHD, so the balance of the fibrinolytic system and the degree of endothelial cell damage will have a slight or serious impact on the pathogenesis of CHD, among which D-D is the most representative.

In this study, the levels of LDL-C, CysC, and D-D in the cases were higher than controls, suggesting that the CHD patients had abnormal expression levels of LDL-C, CysC, and D-D. The CHD patients were further divided, and it was found that the contents of LDL-C, CysC, and D-D in the SAP group, UA group, and AMI group increased successively, suggesting that the levels of LDL-C, CysC, and DD in cases with different clinical types of CHD were different significantly. In addition, the levels of LDL-C, CysC, and D-D were the highest in the three-vessel group and the lowest in the single-vessel group, since the number of lesions can reflect the severity of cases with CHD disease. Once a patient with CHD has multiple lesions in the number of blood vessels, it is very easy to cause myocardial infarction and malignant arrhythmia, which will lead to further deterioration of the patient's condition [13]. The increase in the level of D-D indicates that the activity of fibrinolytic enzyme increases, which increases the viscosity of blood, thereby increasing the aggregation of platelets, resulting in the occurrence of atherosclerotic lumps after the thrombus formed by fibrin and platelets adheres to the blood vessel wall, aggravating the degree of CHD lesions [14]. The more severe the coronary artery lesions, the more severe the patient's myocardial ischemia and hypoxia, resulting in the increase of CysC produced by the body under positive feedback [15]. The logistic regression model showed that high expression levels of LDL-C, CysC, and D-D, male gender, and combined hypertension were risk factors for CHD. Long-term abnormal blood pressure and poor blood pressure control cause the patient's blood vessel wall to be under a condition of high stress and shear force, which increases the production of active substances in the blood vessel wall, which in turn damages the endothelium and its function and eventually leads to blood vessel remodeling. It may interact with endothelial damage caused by high LDL-C, CysC, and DD and jointly promote the process of CHD [16, 17]. Therefore, regular detection of serum LDL-C, CysC, and D-D levels in patients with hypertension plays a significant role in evaluating the degree of target organ damage in cases with essential hypertension and the treatment and prognosis of hypertension [18, 19]. In addition, this study found that the AUC of the combination of LDL-C, CysC, and D-D for the diagnosis of CHD was 0.868, and the sensitivity and specificity were 88.89% and 73.33%, respectively, suggesting that the combination of the above three indicators has good diagnostic performance in CHD.

## 5. Conclusions

In this study, we used monofactor analysis, multifactor analysis, and ROC curve analysis to explore the diagnostic value of LDL-C, CysC, and D-D in CHD. The results showed that LDL-C, CysC, and D-D are highly expressed in CHD patients, and high LDL-C, CysC, and D-D expression levels, male sex, and hypertension are risk factors for CHD. At the same time, the combined detection of LDL-C, CysC, and D-D has good diagnostic performance in CHD, and it can be used as an auxiliary serum index for CHD diagnosis. However, this study has some limitations. First of all, it pays attention to fewer detection indicators, so the research on the risk factors of CHD is not comprehensive. Secondly, the sample size of this study is small, and there may be sampling bias. We will improve our model by including more research objects and exploring more comprehensive laboratory indicators in the next work.

## Figures and Tables

**Figure 1:** The flowchart of patient selection and classification.

**Figure 2:** Comparison of LDL-C levels in CHD patients with different clinical types. Note: compared with SAP group, ^*∗*^*P* < 0.05; compared with UA group, ^*∗∗*^*P* < 0.05.

**Figure 3:** Comparison of CysC levels in CHD patients with different clinical types. Note: compared with SAP group, ^*∗*^*P* < 0.05; compared with UA group, ^*∗∗*^*P* < 0.05.

**Figure 4:** Comparison of D-D levels in CHD patients with different clinical types. Note: compared with SAP group, ^*∗*^*P* < 0.05; compared with UA group, ^*∗∗*^*P* < 0.05.

**Figure 5:** Comparison of LDL-C levels in CHD patients with different lesion branches. Note: compared with SAP group, ^*∗*^*P* < 0.05; compared with UA group, ^*∗∗*^*P* < 0.05.

**Figure 6:** Comparison of CysC levels in CHD patients with different lesion branches. Note: compared with SAP group, ^*∗*^*P* < 0.05; compared with UA group, ^*∗∗*^*P* < 0.05.

**Figure 7:** Comparison of D-D levels in CHD patients with different lesion branches. Note: compared with SAP group, ^*∗*^*P* < 0.05; compared with UA group, ^*∗∗*^*P* < 0.05.

**Figure 8:** ROC diagram of LDL-C, CysC, and D-D and their combination in the diagnosis of CHD.

**Table 1:** Comparison of general clinical data of patients with various clinical kinds of CHD.

Project	Control group (*n* = 30)	Various clinical types of CHD			*F*/*χ*^2^	*P*
		SAP group (*n* = 25)	UA group (*n* = 30)	AMI group (*n* = 35)		
Age (years)	64.07 ± 7.79	62.68 ± 9.03	63.17 ± 7.35	63.34 ± 7.76	0.146	0.932
Gender (male/female)	12/18	12/13	19/11	29/6	14.258	0.003
History of smoking	8 (26.67)	8 (32.00)	8 (26.67)	13 (37.14)	0.811	0.368
High blood pressure	6 (20.00)	13 (52.00)	17 (56.67)	24 (68.57)	18.163	0.000
FPG (mmol/L)	5.73 ± 1.63	5.31 ± 0.92	5.67 ± 1.59	5.84 ± 1.04	0.810	0.491
BUN (mmol/L)	4.84 ± 1.31	4.75 ± 1.40	4.74 ± 0.93	4.77 ± 0.97	0.045	0.987
Cr (*μ*mol/L)	75.00 ± 8.87	75.28 ± 12.35	76.70 ± 14.70	76.38 ± 12.37	0.136	0.938
TC (mmol/L)	4.65 ± 0.99	4.39 ± 0.56	4.31 ± 0.85	4.37 ± 0.91	0.932	0.428
TG (mmol/L)	1.45 ± 0.63	1.41 ± 0.41	1.45 ± 0.60	1.42 ± 0.67	0.034	0.991

**Table 2:** Relationship between the number of different lesions in cases and general clinical data.

Project	Control group (*n* = 30)	Different clinical types of CHD			*F*	*P*
		SAP group (*n* = 25)	UA group (*n* = 30)	AMI group (*n* = 35)		
Age (years)	64.07 ± 7.79	63.68 ± 9.01	63.47 ± 7.38	63.42 ± 6.71	0.041	0.989
Gender (male/female)	12/18	24/10	11/19	21/5	17.115	0.001
History of smoking	8 (26.67)	9 (26.47)	7 (23.33)	5 (19.23)	0.558	0.906
High blood pressure	6 (20.00)	19 (55.88)	16 (53.33)	19 (73.08)	16.942	0.000
FPG (mmol/L)	5.73 ± 1.63	5.50 ± 1.44	5.75 ± 1.26	5.78 ± 1.31	0.261	0.853
BUN (mmol/L)	4.84 ± 1.31	4.89 ± 0.92	4.81 ± 1.01	4.86 ± 0.95	0.032	0.992
Cr (*μ*mol/L)	75.00 ± 8.87	75.41 ± 12.40	75.86 ± 6.16	75.87 ± 7.44	0.060	0.981
TC (mmol/L)	4.65 ± 0.99	4.60 ± 0.96	4.63 ± 0.73	4.66 ± 0.86	0.027	0.994
TG (mmol/L)	1.45 ± 0.63	1.46 ± 0.41	1.47 ± 0.22	1.49 ± 0.46	0.040	0.989

**Table 3:** Comparison of LDL-C, CysC, and D-D levels between cases and controls ($\bar{x}\pm \text{s}$).

Group	LDL-C (mmol/L)	CysC (mg/L)	D-D (mg/L)
Control group (*n* = 30)	2.25 ± 0.77	1.08 ± 0.42	0.98 ± 0.57
CHD group (*n* = 90)	3.27 ± 0.72	1.43 ± 0.52	1.54 ± 0.50
*t*	6.604	3.338	5.127
*P*	0.000	0.001	0.000

**Table 4:** Comparison of LDL-C, CysC, and D-D levels in patients with various clinical types of CHD ($\bar{x}\pm \text{s}$).

Group	LDL-C (mmol/L)	CysC (mg/L)	D-D (mg/L)
SAP group (*n* = 25)	2.66 ± 0.71	1.08 ± 0.45	1.14 ± 0.63
UA group (*n* = 30)	3.22 ± 0.63^a^	1.38 ± 0.53^a^	1.48 ± 0.46^a^
AMI group (*n* = 35)	3.70 ± 0.32^ab^	1.71 ± 0.35^ab^	1.89 ± 0.45^ab^
*F*	25.398	14.894	16.193
*P*	0.000	0.000	0.000

*Note.* Compared with SAP group, ^a^*P* < 0.05; compared with UA group, ^b^*P* < 0.05.

**Table 5:** Comparison of LDL-C, CysC, and D-D levels in CHD patients with different number of lesions ($\bar{x}\pm \text{s}$).

Group	LDL-C (mmol/L)	CysC (mg/L)	D-D (mg/L)
Single-branch group (*n* = 34)	2.70 ± 0.37	1.11 ± 0.45	1.23 ± 0.59
Double-branch group (*n* = 30)	3.30 ± 0.41^a^	1.45 ± 0.53^ab^	1.58 ± 0.35^a^
Three-branch group (*n* = 26)	3.98 ± 0.51^ab^	1.83 ± 0.41^ab^	1.90 ± 0.52^ab^
*F*	66.174	17.494	13.339
*P*	0.000	0.001	0.000

*Note.* Compared with the single-branch group, ^a^*P* < 0.05; compared with the double-branch group, ^b^*P* < 0.05.

**Table 6:** Analysis of risk factors affecting the occurrence of CHD.

Independent variable	*β*	SE	Wald *χ*^2^	OR	95% CI	*P*
LDL-C	0.152	0.047	10.459	1.164	1.062–1.276	0.001
CysC	0.300	0.128	5.493	1.350	1.050–1.735	0.020
D-D	0.205	0.058	12.493	1.228	1.096–1.375	0.005
Male	0.241	0.114	4.469	1.273	1.018–1.591	0.035
Combined hypertension	0.158	0.074	4.559	1.171	1.013–1.354	0.033

**Table 7:** Analysis of the efficacy of LDL-C, CysC, and D-D in the diagnosis of CHD.

Indicator	Cutoff	AUC	Youden index	Sensitivity	Specificity	95% CI	*P*
LDL-C	>2.71	0.829	0.622	82.22	80.00	0.749–0.891	0.000
CysC	>1.46	0.688	0.367	46.67	90.00	0.597–0.769	0.000
D-D	>0.80	0.776	0.500	86.67	63.33	0.691–0.847	0.000
Joint detection	—	0.868	0.622	88.89	73.33	0.794–0.923	0.000

## Data Availability

The data used to support the findings of this study are available from the corresponding author upon request.
